The article "Chitosan-Based Nanocapsules as a Delivery System of Hydrophobic Carnosic Acid, A Model Neuroprotective Drug" was published in 2024. Journal: Nanotechnol Sci Appl.

# Chitosan-Based Nanocapsules as a Delivery System of Hydrophobic Carnosic Acid, A Model Neuroprotective Drug

**DOI:** 10.2147/NSA.S490372

**Published:** 2024-12-20

**Authors:** Joanna Odrobińska-Baliś, Magdalena Procner, Kinga Krużel, Magdalena Regulska, Monika Leśkiewicz, Dorota Duraczyńska, Szczepan Zapotoczny, Władysław Lasoń, Krzysztof Szczepanowicz

**Affiliations:** 1 Jerzy Haber Institute of Catalysis and Surface Chemistry, Polish Academy of Sciences, Krakow, Poland; 2 Maj Institute of Pharmacology Polish Academy of Science, Krakow, Poland; 3 Faculty of Chemistry, Jagiellonian University, Krakow, Poland

**Keywords:** polysaccharide nanocapsules, modified chitosan, carnosic acid, neuroprotection

## Abstract

**Introduction:**

Since the population of Europe is rapidly aging, the number of cases of neurodegenerative diseases sharply increases. One of the most significant limitations of current neurodegenerative disease treatment is the inefficient delivery of neuroprotective drugs to the affected part of the brain. One of the promising methods to improve the pharmacokinetic and pharmacodynamic properties of antioxidants is their encapsulation in nanocarriers.

**Materials and Methods:**

Encapsulation of carnosic acid into a chitosan-based nanoparticle system with ultrasound-assisted emulsification process was developed. The physicochemical properties (size, stability, concentration of nanoparticles) of obtained nanocapsules were analyzed. Also, the cytotoxicity and neuroprotective effect in SH-SY5Y cells exposed to toxic concentration of H_2_O_2_ of the obtained nanoparticles were evaluated in vitro.

**Results and Discussion:**

The capsules with diameters between 90 and 150 nm and long-term stability were obtained. Cytotoxicity tests of empty capsules indicate that observed toxic effects were concentration dependent and lower concentrations (dilution above 500×) can be considered as safe for tested cells. Our study also indicates that encapsulation of carnosic acid decreased the cytotoxicity of empty nanocapsules and can efficiently protect SH-SY5Y cells from factors causing cell destruction. In addition, the neuroprotective efficacy of carnosic acid loaded nanocapsules was also demonstrated in SH-SY5Y cells exposed to toxic concentration of H_2_O_2_. The designed nanoparticles appear to possess sufficient biocompatibility to deserve their further evaluation in in vivo models.

## Introduction

Since the population of Europe is rapidly aging the number of cases of neurodegenerative diseases such as stroke, Alzheimer’s and Parkinson’s sharply increases. Two-thirds of strokes occurred generally in those over 65 years old^1^ that is why prevention and treatment of stroke-related brain damage and neurodegenerative diseases are growing problems of contemporary medicine. Understanding the pathophysiological mechanisms associated with neuronal injury due to stroke is of significant importance. Oxidative stress, a pathologic process resulting from an imbalance between production and accumulation of oxygen reactive species (ROS) in cells and tissues, has been considered as one of the major mechanisms for inducing neuronal damage by ischemia. Oxidative stress participates in stroke-related activation of cell death/survival signal pathways, mitochondrial dysfunction, inflammatory response, and blood–brain barrier (BBB) disruption.^2^,^3^ Of note, the removal of pathologically produced free radicals by natural or synthetic antioxidants has been proposed for a long time as a feasible neuroprotective strategy^4^ Although natural antioxidants show high activity in the scavenging of free radicals, their bioavailability is constricted by low absorption and poor stability. Indeed, one of the most significant limitations of current neurodegenerative disease treatment is the inefficient delivery of neuroprotective drugs to the affected part of the brain. The blood–brain barrier (BBB) is permeable to small (<1000 Da), lipophilic molecules only and limits the transfer to the brain of most drugs, including imaging contrast agents, and macromolecular compounds.^5^,^6^ To this end, nanotechnology offers new solutions to improve therapies for central nervous system (CNS) disorders with the use of drug nanocarriers which enable neuroprotective drugs to reach and maintain their therapeutic concentration in the brain. One of the promising methods to improve the pharmacokinetic and pharmacodynamic properties of antioxidants is their encapsulation in nanocarriers. Nanocarriers have attracted significant interest in the delivery to CNS due to their unique properties and multifunctionalities.^7^ By tuning physicochemical properties such as size, shape, surface charge, and coating ligands, the transport efficiency to CNS could be enhanced.^8^ Several excellent review papers have been published on strategies for NP-mediated brain drug delivery, including a discussion on the physicochemical properties of nanocarriers.^8–12^ Herein, based on previous research, we chose carnosic acid^13^ as a naturally occurring antioxidant which is responsible for 90% of the antioxidant properties of rosemary extract.^14^ Carnosic acid (CA) apart from being a strong antioxidant with a neuroprotective effect on neuronal cells^15^ possesses also a vast array of beneficial properties including antimicrobial, anti-inflammatory, and anticarcinogenic activities.^16–18^ CA has poor water solubility and is unstable, particularly in solvents, and is easily degraded by the effects of light and oxygen exposure.^19^,^20^ Since nano and microcapsules are suitable for poorly water-soluble substances, we encapsulated CA in an oil core polysaccharide nanocapsules to improve its physicochemical stability and aqueous solubility. Specifically, we focused on the modified/functionalized chitosan with charged hydrophilic backbone and hydrophobic side chains for the stabilization of oil droplets for designing more robust delivery systems.^21–23^ Such polymers provide enhanced stabilization of nanoemulsions due to anchoring in the oil droplet by hydrophobic arms and electrostatic repulsions between the charged capsule shells.

The article "Chitosan-Based Nanocapsules as a Delivery System of Hydrophobic Carnosic Acid, A Model Neuroprotective Drug" was published in 2024. Journal: Nanotechnol Sci Appl.

In the present work, we developed a novel approach to encapsulate CA into a chitosan-based nanoparticle system. Three types of oil liquid cores of hydrophobically modified derivatives of chitosan-based nanocapsules were designed and tested. Since the biosafety is crucial for designing nanoparticles for biomedical applications, the potential cytotoxicity of the obtained nanocapsules was evaluated in vitro. Further in vitro study showed neuroprotective effect of nanoencapsulated CA, which suggests that the proposed nanocapsules may also serve as a convenient drug delivery platform for other neuroprotective agents. However, this assumption has to be confirmed in future studies using in vivo models.

## Materials and Methods

### Materials for Nanocapsules Preparation

Sodium chloride (NaCl, Sigma-Aldrich)), oleic acid (OA, Ph, Eur., 65.0–88.0% (GC), Sigma-Aldrich), corn oil (CORN, Sigma-Aldrich), MCT oil (MCT, MCT Oil based on Coconut Oil, Gustav Heess Sp. z o.o)., perylene (Pe, gold label, 99.9%, Sigma-Aldrich), hydrogen peroxide (30% solution, p.a., Avantor Performance Material Poland S.A)., and sulfuric acid (H_2_SO_4_, 96%, Chempur), chitosan (LMW, Mw < 150,000 g/mol, Sigma-Aldrich), glycidyltrimethylammonium chloride (GTMAC, Sigma-Aldrich), acetone (p.a., Chempur), N-dodecyl aldehyde (92%, Sigma-Aldrich), sodium cyanoborohydride (95%, Sigma-Aldrich), diethyl ether (p.a., Chempur), carnosic acid (ChemNorm Biotech Co. Ltd). Deionized water was used to prepare all the solutions. All materials were used without further purification.

### Materials for Cell Culture and Cytotoxicity Tests

The human SH-SY5Y neuroblastoma cell culture was obtained from the American Type Culture Collection (ATCC, CRL-2266, Manassas, VA, USA). Dulbecco’s Modified Eagle Medium (DMEM), 0.25% Trypsin-EDTA solution, Penicillin–Streptomycin mixture (10,000 U/mL), heat-inactivated fetal bovine serum (FBS), and N-2 supplement were purchased from Gibco (Life Technologies Ltd). Triton X-100 solution and hydrogen peroxide solution 30% (w/w) in H_2_O were obtained from Sigma-Aldrich Chemie GmbH. Cell Proliferation Reagent WST-1 and Cytotoxicity Detection Kit (LDH) were provided by Roche Diagnostics GmbHAll materials were used without further purification. All reported concentrations are the final values obtained after mixing and diluting the reactants.

The article "Chitosan-Based Nanocapsules as a Delivery System of Hydrophobic Carnosic Acid, A Model Neuroprotective Drug" was published in 2024. Journal: Nanotechnol Sci Appl.

### Modification of Chitosan

A cationic amphiphilic chitosan derivative (CChitC12) containing both quaternary ammonium groups and n-dodecyl groups was synthesized according to the slightly modified procedure described previously by Bulwan et al.^24^ Briefly, 3.4 g of chitosan was dissolved in 1% acetic acid to prepare 2% (w/v) chitosan solution. Then, 15 mL of GTMAC was added. The reaction mixture was kept at 70 °C for 24 h. The resulting polymer was purified by precipitation into the 1:1 (v/v) cooled mixture of acetone and methanol. The precipitate was centrifuged, washed with acetone and then with ethanol (3 times per solvent). To remove unreacted residues, the precipitate was dissolved in deionized water and centrifuged. The polymer from the supernatant was then precipitated in a mixture of cooled acetone and ethanol (4:1, v/v). The precipitate was washed with ethanol, centrifuged and dissolved in deionized water. The obtained mixture was dialyzed against water for 7 days and freeze-dried. The final product was characterized by ^1^H NMR spectroscopy to determine the degree of substitutions DS, which was 78 mol-% for quaternary ammonium groups and 3.5 mol-% for dodecyl groups.

### Preparation of Core-Shell Chitosan Based Nanocapsules Loaded with Carnosic Acid

An ultrasound-assisted emulsification process was applied to obtain chitosan-based capsules according to previously described procedures.^21^,^25^,^26^ Briefly, the aqueous solution of (CChitC12) (1 g/L in 0.15 M NaCl) was mixed with the appropriate oil (OA, CORN or MCT) in a 1000:5 (v/v) ratio. The mixture was homogenized using a vortex shaker and then sonicated for 16 min (8 min sonication, 6 min break, 8 min sonication) at room temperature with the ultrasonic generator (Sonics Processor VCX750, Sonics & Materials, Inc., Newton, USA) working in pulse mode (pulse time: 1s, break time: 2s) with 45% of the maximum amplitude, 600 W. For drug-loaded nanocapsules, CA was dissolved in corn oil, MCT oil or oleic acid, and the solution was further used as an oil phase in the process of the capsules preparation. The concentration of CA in the nanocapsules oil cores (per 1 mL of capsules suspension) was ca. 0.1 mg/mL in corn oil, 0.05mg/mL in MCT oil and 0.2 mg/mL in oleic acid.

The article "Chitosan-Based Nanocapsules as a Delivery System of Hydrophobic Carnosic Acid, A Model Neuroprotective Drug" was published in 2024. Journal: Nanotechnol Sci Appl.

### Size, Size Distribution and Zeta Potential Measurements

A Malvern Zetasizer Nano ZS instrument working at a 173° detection angle was used for dynamic light scattering (DLS) measurements. The measurements of hydrodynamic diameter were performed at 22°C, and the reported data represent the averages from three series of measurements (10−100 runs each) and their standard deviations. General purpose mode and size distribution by number were used as the distribution analysis algorithm. ζ-potential was determined also with Malvern Zetasizer Nano ZS apparatus using laser Doppler velocimetry (LDV). Moreover, the Malvern NanoSight NS300 instrument was used for nanoparticle tracking analysis (NTA) to characterize size and estimate the quantity of obtained nanocapsules. Measurements were performed using light scatter from the 405 nm violet laser. Data represent the averages from three series of measurements (6 runs each).

### Visualization by Confocal Microscopy and Scanning Electron Microscopy

The fluorescent dye, perylene, was dissolved in corn oil, MCT oil and oleic acid. The concentration of perylene in the nanocapsules cores was *ca*. 0.004 M. The solution was further used as an oil phase in the process of the preparation of dye-loaded nanocapsules. Confocal microphotographs were collected using a Nikon Ti-E inverted microscope with an objective Plan Apo 100×/1.4 oil DIC and a Nikon A1 confocal system.

For the scanning electron microscopy (SEM), a droplet of capsule suspension was deposited on the silicon wafer that was firstly cleaned carefully using a piranha solution (a mixture of 96% H_2_SO_4_ and 30% H_2_O_2_ solutions with a volume ratio of 1:1) and dried in a stream of argon. To avoid the presence of NaCl crystals in SEM images, capsules were prepared in deionized water instead of NaCl solution. Scanning electron micrographs were collected by a JEOL JSM-7500F instrument (JEOL, Tokyo, Japan).

### SH-SY5Y Cell Culture and Treatment

The human SH-SY5Y neuroblastoma cells were grown in DMEM (Dulbecco’s Modified Eagle Medium, high glucose) supplemented with 10% (v/v) heat-inactivated FBS and 1% (v/v) penicillin–streptomycin mixture^27^ in plastic T75 culture flasks. The cells were incubated at 37°C under saturated humidity conditions (95% air, 5% CO_2_). When cells have reached 80% confluence they were trypsinized using 0.05% Trypsin/EDTA solution, counted manually (Bürker chamber) and seeded at a density of 5 × 10^4^ cells per well in 100 µL of a supplemented medium into 96-well plates. Next, the plates were incubated for 24–48 h to ensure optimal cell growth. Cell treatment was carried out 24 h after replacing the culture medium, with serum-free DMEM containing antibiotics and 1% (v/v) N-2 supplement. Subsequently, SH-SY5Y cells were treated in the presence of 10 µL appropriately diluted chitosan nanoparticles (final dilutions in the culture medium 10×, 20×, 40×, 80×, 100×, 200× and 500×, respectively, depending on the type of sample) to assess the biosafety results. Then, the plates were maintained under standard conditions for 24 hours. For neuroprotection experiments, SH-SY5Y cells were pre-treated with different concentrations of three types of CA-loaded chitosan nanocapsules. After 30 minutes of incubation, hydrogen peroxide was added in two dilutions (final concentrations 0.375 mm and 0.5 mm) to induce cell damage. In all described experiments, H_2_O_2_ and chitosan nanocapsules were freshly diluted in Mili-Q distilled water or 15 mm NaCl solution, respectively. The control cultures were supplemented with 10 µL of vehicle (15 mm NaCl solution). To assess the control for maximum cell membrane damage, the cells from selected wells were lysed with 1 µL of Triton X-100.

The article "Chitosan-Based Nanocapsules as a Delivery System of Hydrophobic Carnosic Acid, A Model Neuroprotective Drug" was published in 2024. Journal: Nanotechnol Sci Appl.

### Cytotoxicity Assay

The potential cytotoxicity of chitosan nanocapsules was evaluated by measuring the level of lactate dehydrogenase (LDH) release from treated cells to the culture medium. The LDH release is strictly correlated with cell membrane destruction and therefore serves as a reliable marker of cell death. Twenty-four hours after cell treatment, the 50 µL of cell-free supernatants from each well were transferred to a fresh 96-well plate, mixed with LDH reagent from Cytotoxicity Detection Kit according to the supplier’s instructions and incubated at room temperature for 10–15 minutes. The absorbance, for all samples, at wavelength 490 nm was measured using the multi-well plate-reader (Infinite^®^ M200 PRO, Tecan, Switzerland). The absorbance of background from wells with a mixture of pure medium and LDH reagent was subtracted from each measurement. Obtained values were normalized to the level of LDH released from vehicle-treated cells and expressed as a percentage of control ± SEM established from at least 4 independent experiments with 3–5 replicates each.

### Cell Viability Assay

The assessment of cell viability in SH-SY5Y cells exposed to different dilutions of chitosan nanocapsules was evaluated by the WST-1 assay using a standard manufacturer’s protocol. The 5 µL of WST-1 reagent (4-[3-(4-Iodophenyl)-2-(4-nitro-phenyl)-2H-5-tetrazolio]-1,3-benzene sulfonate) was added to each well and plates were incubated at 37°C. Subsequently, the absorbance of each sample was determined after 30 and 60 minutes of incubation with a multi-well plate-reader Infinite^®^ M200 PRO (Tecan, Switzerland) at 440 nm and 630 nm (measurement and reference wavelength, respectively). Before further data analysis, the blank value (cells treated with 1 µL of Triton X-100 for 15 min) was subtracted from the data calculated as differences between values of measurement and reference wavelength. Obtained results were normalized to the control cells and presented as a percentage of control ± SEM determined from at least 4 independent experiments with 3 to 5 replicates each.

The article "Chitosan-Based Nanocapsules as a Delivery System of Hydrophobic Carnosic Acid, A Model Neuroprotective Drug" was published in 2024. Journal: Nanotechnol Sci Appl.

### Statistical Analysis

Data after normalization to the control groups were analyzed using the Statistica 13.3 software (StatSoft Inc., Tulsa, OK, USA). The differences between groups were calculated using the analysis of variance (one-way ANOVA) and *post-hoc* Duncan’s test. Statistical results were expressed as the mean ± SEM from at least four independent experiments. Differences were considered significant at the p <0.05.

## Results

### Preparation and Physicochemical Properties of Nanocapsules with CA

Chitosan-based nanocapsules with encapsulated CA in the core were obtained in an ultrasound-assisted direct homogenization process by simple mixing of proper oil phase (oleic acid, corn oil, MCT oil) containing CA with an aqueous solution of amphiphilic chitosan derivative (Figure 1). Concentration CA was chosen on the basis of its highest solubility in the oil phases reached in our laboratory, ie, 40 g/l for oleic acid, 20 g/l for corn oil, 10 g/l for MCT oil.

**Figure 1:** Scheme of preparation of chitosan-based capsules with incorporated CA.

The formation of the nanocapsules was followed using dynamic light scattering (DLS), and nanoparticle tracking analysis (NTA). For all of the oils for drug-loaded as well as empty capsules, the diameter between 90 and 150 nm and low PDI (below 0.3) were observed just after sonication (Figure 2- week 0). The measured absolute values of zeta potential were ~ +20-25 mV which did not satisfy the electrostatic stability criterion for colloidal systems (|ζ|>30 mV), therefore we tested the stability of chitosan-based nanocapsules by monitoring their size and zeta potential during prolonged storage at 4 °C up to 4 weeks for empty and 8 weeks for CA loaded capsules (Figure 2). The values of measured parameters did not significantly change in time, suggested good stability of prepared nanocapsules over time. Some small fluctuations in the size of hydrodynamic diameters for CA-loaded capsules with corn oil as the core can be observed after 1 week of storage; however, it can be interpreted as an artifact since this anomaly disappeared in the next measurements, ie, after 2 or more weeks.

**Figure 2:** (**A**) - Number-weighted distribution of diameters of the studied chitosan-based (CH) empty capsules with respected oil cores (CH-MCT, CH-OA, CH-CORN) as determined by DLS measurements during 4 week storage time and capsules with encapsulated CA during 8 week storage time (CA-CH-MCT, CA-CH-OA, CA-CH-CORN). (**B**) - Number-weighted average hydrodynamic diameters of studied empty capsules as determined by DLS measurements during 4 week storage time and capsules with encapsulated CA during 8 week storage. (**C**)- Zeta potential values of the studied empty capsules as determined by DLS measurements during 4 week storage time and capsules with encapsulated CA during 8 week storage time. Error bars represent standard deviations of 3 measurements.

The article "Chitosan-Based Nanocapsules as a Delivery System of Hydrophobic Carnosic Acid, A Model Neuroprotective Drug" was published in 2024. Journal: Nanotechnol Sci Appl.

Moreover, the sizes of the hydrodynamic diameters of the capsules measured using the DLS method coincide quite well with the sizes of the hydrodynamic diameters measured using the NTA method. The comparison is summarized in the table where results of particle concentration measurements were also collected (Table 1).

**Table 1:** Comparison of Size of Hydrodynamic Diameter of Capsules Measured with DLS Method and NTA Method and Capsules Concentration (Data Collected Two Weeks After Capsules Preparation)

Capsules	PDI	SIZE [nm]	ZETA [mV]	NTA Mode [nm]	Particles Concentration [Particles/mL]
**CH-CORN**	0.19	128 ± 5	21 ± 1	182	(2.84±0.08)∙10^11^
**CH-MCT**	0.15	140 ± 5	22 ± 1	174	(1.23±0.03)∙10^12^
**CH-OA**	0.14	137 ± 8	22±3	136	(1.75±0.11)∙10^11^
**CA-CH-CORN**	0.19	123 ± 52	21 ± 2	141	(1.85±0.10)∙10^11^
**CA-CH-MCT**	0.15	110 ± 3	17±1	125	(2.35±0.25)∙10^11^
**CA-CH-OA**	0.11	115 ± 2	20 ± 1	120	(3.61±0.21)∙10^11^

SEM images (Figure 3) show collapsed polymer coatings in the shape of blood cells with a clearly visible place of the capsule core with diameters between 100 and 200 nm (empty capsules with oleic acid core), despite SEM microscopy not being the best method for imaging liquid-core capsules due to the lack of an aqueous environment and the presence of a vacuum cause the capsules to collapse.

**Figure 3:** SEM images of capsules with oleic acid core.

The ability of encapsulation of hydrophobic compounds was examined using a fluorescent probe, ie, perylene. The confocal micrographs, shown in Figure 4, confirmed that the perylene, which is only sparingly soluble in water and has negligible fluorescence in an aqueous solution was located in the hydrophobic cores of the capsules. Furthermore, no variations in particle size were observed which indicates that the encapsulation did not affect the morphology of the capsules and did not generate a tendency to capsule aggregation.

**Figure 4:** Confocal micrographs of chitosan-based nanocapsules templated on (**A**) MCT oil (**B**) oleic acid (**C**) corn oil cores with encapsulated perylene using λ_ex_ = 405 nm and DAPI filter.

The article "Chitosan-Based Nanocapsules as a Delivery System of Hydrophobic Carnosic Acid, A Model Neuroprotective Drug" was published in 2024. Journal: Nanotechnol Sci Appl.

### The Effect of Chitosan Nanoparticles on in vitro Cytotoxicity

Evaluation of biosafety is crucial for designing nanoparticles that can be potentially used as neuroprotective drug delivery systems. Therefore, the effect on in vitro cytotoxicity and viability of human neuroblastoma cells exposed to all types of nanocapsules was examined via LDH and WST-1 assays. First, SH-SY5Y cells were incubated with different dilutions of chitosan nanocapsules (empty and loaded with CA). After 24 h, the level of lactate dehydrogenase released into the culture medium was measured to perform a cell death assessment. At the beginning, we examined the empty chitosan nanocapsules in different dilutions in human neuroblastoma cell cultures. We observed that all three types of the tested nanocapsules exerted a strong toxic effect on the cells as reflected by an increase in LDH activity after 24 h of treatment (Figure 5A). Only the capsules based on corn oil in 500× dilution did not influence lactate dehydrogenase release as compared to control values. This result clearly indicates that empty chitosan nanocapsules affect the cell membrane integrity. Moreover, the viability of the SH-SY5Y cells exposed to empty nanocapsules was decreased almost for all examined dilutions (Figure 5B). The observed toxic effects were concentration-dependent, and dilution above 500× can be considered as safe for tested cells. At this point, it is worth emphasizing that cytotoxicity in the lowest applied dilutions may result from positive surface charge of chitosan nanocapsules. Based on the literature, many experiments/studies clearly indicate the influence of nanoparticles’ physicochemical properties on therapeutic bioavailability, cytotoxicity, cellular uptake and internalization.^28^ Many studies showed that the cytotoxicity of nanoparticles and mechanism of cell death are strongly affected by their surface charge, where the cationic ones were found to be more toxic than anionic or neutral NPs.^29–32^ However, the particle size and surface charge have a significant impact on transport processes through biological barriers or lipid bilayer.^33^,^34^ It is believed that positive charge of the surface may promote higher uptake (by endocytosis or by direct penetration) via electrostatic interactions with negatively charged cell membrane (anionic parts/groups of biomolecules such as proteins, phospholipids etc.);^28^,^29^,^31^,^35–43^ however, the cationic character may also cause rapid NPs release from therapeutic targets.^44^,^45^ Nevertheless, we would like to emphasize that the presented toxicity results do not disqualify our nanocapsules as promising for further studies – even for 500× dilution for empty NCs, concentrations remain on significant level and may be considered as therapeutic valuable.

The article "Chitosan-Based Nanocapsules as a Delivery System of Hydrophobic Carnosic Acid, A Model Neuroprotective Drug" was published in 2024. Journal: Nanotechnol Sci Appl.

**Figure 5:** The effect of chitosan nanocapsules in different dilutions on the LDH release (**A**) and cell viability (**B**) of human neuroblastoma SH-SY5Y cells. The LDH release and WST-1 assays were performed after 24 h of treatment with appropriate diluted NCs. The control cells were supplemented with distilled water as vehicle. The data were normalized to the vehicle-treated cells and expressed as the mean (in percent) ± SEM from at least 4 independent experiments with 3–5 replicates. *p < 0.05 vs vehicle-treated cells.

CA-loaded nanocapsules were also examined based on their in vitro cytotoxicity and viability in human neuroblastoma cells. It is worth noting that we did not find any pronounced cell damaging effect of three types of CA-loaded nanocapsules at dilutions 100–500× as evidenced by LDH assays (see Figure 5A). Only the 10× dilutions after 24 h increased cell damage in the conducted experiments. These results were confirmed by the WST-1 test, in which all samples 10× diluted decreased cell viability by more than 40% of the control value (Figure 5B); however, we also observed that nanocapsules formed with corn oil, and oleic acid were slightly toxic in higher (100×) dilution (Figure 5B). Comparing the three 10× diluted samples with each other, it is worth highlighting that OA-based nanocapsules showed the highest toxicity in both applied assays. It can be attributed to the previously observed toxicity of oleic acid if efficiently delivered to cells such as in nanocapsules.^23^ In contrast, the MCT oil-based sample with a lower concentration of CA was the safest for SH-SY5Y cells.

Overall, the data obtained in neuroblastoma cell cultures showed a pronounced difference between empty and CA-loaded nanocapsules in their biosafety. Such discrepancy may be correlated with the impact of CA itself. Our study indicates that CA decreased the cytotoxicity of three examined nanocapsules and can efficiently protect SH-SY5Y cells from factors causing cell destruction. The assumption that carnosic acid effectively reduced toxic effects of chitosan nanocapsules may be associated with its strong antioxidant and neuroprotective properties. Our in vitro results are in line with other literature reports showing that CA has the ability to protect different types of cell cultures, ie, human neuroblastoma cells and primary neuronal cells from various types of cell damage.^13^,^46–50^

### The Effect of Chitosan Nanoparticles on H_2_O_2_-Induced Cell Damage

The protective effect of CA incorporated into chitosan-based nanocapsules was further confirmed by testing three types of CA-loaded nanocapsules CA-CH-CORN, CA-CH-MCT and CA-CH-OA against oxidative stress-induced cell damage. Human neuroblastoma cells were treated with two concentrations (0.375 mm or 0.5 mm) of hydrogen peroxide for 24 h and afterward, LDH and WST-1 assays were performed. Experimental data showed that hydrogen peroxide alone in both concentrations intensively increased the level of released LDH after cell treatment (Figure 6). However, CA-loaded chitosan nanocapsules formed with corn and MCT oil in 200× dilution (and sometimes 500× dilution, see Figure 6) substantially diminished LDH leakage from the cells to the culture medium by more than 20% (compared to the effect of H_2_O_2_ in appropriate concentration alone). These results were also confirmed in the cell viability experiments in which such nanocapsules meaningly protected SH-SY5Y cells against H_2_O_2_-evoked neuronal death in the above-mentioned dilutions (Figure 6). The cell loss after 24 h exposition to chitosan nanocapsules was slightly reduced compared to untreated cells, while hydrogen peroxide alone at both concentrations decreased cell viability by about 20–35%. As shown in Figure 6, only 500× diluted CA-CH-OA sample decreased LDH release by about 30% compared with 0.5 mm H_2_O_2_ treated cells. We also observed that such nanocapsules in experiments with higher hydrogen peroxide concentration slightly enhance cell viability up to more than 80%, although these data were not statistically significant. These results clearly indicate that among the three types of CA-loaded chitosan nanocapsules, the corn and MCT oil ones displayed much higher neuroprotective efficiency than nanocapsules based on oleic acid, as detected in both LDH and WST-1 assays.

The article "Chitosan-Based Nanocapsules as a Delivery System of Hydrophobic Carnosic Acid, A Model Neuroprotective Drug" was published in 2024. Journal: Nanotechnol Sci Appl.

**Figure 6:** The effect of CA-CH-CO (**A** and **B**), CA-CH-MCT (**C** and **D**), CA-CH-OA (**E** and **F**) chitosan nanoparticles in different dilutions on the LDH release (**A, C**, and **E**) and cell viability (**B, D** and **F**) of human neuroblastoma SH-SY5Y cells alone and against H_2_O_2_-induced cell damage. The LDH release and WST-1 assays were performed after 24 h of treatment with appropriate diluted NPs or NPs and hydrogen peroxide (concentration 0.375 mm or 0.5 mm). The control cells were supplemented with distilled water as a vehicle or a suitable volume of H_2_O_2_ as a negative control to define the maximum cell damage caused by hydrogen peroxide. The data were normalized to the vehicle-treated cells and expressed as the mean (in percent) ± SEM from at least 4 independent experiments with 3–5 replicates. *p < 0.05 vs vehicle-treated cells; #p < 0.05 vs H_2_O_2_-treated cells at appropriate dilution.

## Conclusions

As the population of Europe is rapidly aging, the design of neuroprotective compound delivery systems has been recently considered as a major challenge for modern nanomedicine. CA, which naturally occurs in rosemary extract, is an antioxidant with an attributed neuroprotective effect on neuronal cells but unfortunately it displays poor solubility in water and poor stability. To address this problem, polysaccharide-based nanocapsules with three different types of liquid oil cores were developed as carriers of hydrophobic neuroprotective compounds. Obtained nanoparticles were characterized by small sizes of hydrodynamic diameters, high stability during prolonged storage confirmed by dynamic light scattering, nanoparticle tracking analysis and zeta potential measurements. The nanocapsules showed cytotoxicity only in the highest doses, and it decreases in concentration-dependent manner in neuroblastoma cell cultures. The comparison of biosafety data for all tested samples revealed the neuroprotective potency of CA-loaded nanocapsules. Furthermore, the neuroprotective efficacy of CA-loaded nanocapsules was also demonstrated in SH-SY5Y cells exposed to toxic concentration of H_2_O_2_. Of note, among the three types of CA-loaded chitosan nanocapsules, the corn and MCT oil ones displayed much higher neuroprotective efficacy than nanocapsules based on oleic acid. Overall, the designed NPs appear to possess sufficient biocompatibility to deserve their further evaluation in in vivo models. Our results also indicate that chitosan-based nanocapsules with oil-liquid cores possess favourable physicochemical properties, and they are promising candidate for nano-delivery systems for hydrophobic/lipophilic neuroprotective compounds.

## References

[1] Feigin VL, Forouzanfar MH, Krishnamurthi R, et al. Global and regional burden of stroke during 1990-2010: findings from the global burden of disease study 2010. *Lancet*. 2014;383(9913):245–254. doi:10.1016/s0140-6736(13)61953-424449944 PMC4181600

[2] Chen H, Yoshioka H, Kim GS, et al. Oxidative stress in ischemic brain damage: mechanisms of cell death and potential molecular targets for neuroprotection. *Antioxid Redox Signal*. 2011;14(8):1505–1517. doi:10.1089/ars.2010.357620812869 PMC3061196

[3] Feng S, Yang M, Liu S, He Y, Deng S, Gong Y. Oxidative stress as a bridge between age and stroke: a narrative review. *J Intensive Med*. 2023;3(4):313–319. doi:10.1016/j.jointm.2023.02.00238028635 PMC10658045

[4] Green AR, Ashwood T. Free radical trapping as a therapeutic approach to neuroprotection in stroke: experimental and clinical studies with NXY-059 and free radical scavengers. *Curr Drug Targets CNS Neurol Disord*. 2005;4(2):109–118. doi:10.2174/156800705354415615857295

The article "Chitosan-Based Nanocapsules as a Delivery System of Hydrophobic Carnosic Acid, A Model Neuroprotective Drug" was published in 2024. Journal: Nanotechnol Sci Appl.

[5] Tam VH, Sosa C, Liu R, Yao N, Priestley RD. Nanomedicine as a non-invasive strategy for drug delivery across the blood brain barrier. *Int J Pharm*. 2016;515(1–2):331–342. doi:10.1016/j.ijpharm.2016.10.03127769885

[6] Furtado D, Björnmalm M, Ayton S, Bush AI, Kempe K, Caruso F. Overcoming the blood–brain barrier: the role of nanomaterials in treating neurological diseases. *Adv Mater*. 2018;30(46). doi:10.1002/adma.20180136230066406

[7] Qiao R, Fu C, Forgham H, et al. Magnetic iron oxide nanoparticles for brain imaging and drug delivery. *Adv Drug Deliv Rev*. 2023;197:114822. doi:10.1016/j.addr.2023.11482237086918

[8] Saraiva C, Praça C, Ferreira R, Santos T, Ferreira L, Bernardino L. Nanoparticle-mediated brain drug delivery: overcoming blood-brain barrier to treat neurodegenerative diseases. *J Control Release*. 2016;10(235):34–47. doi:10.1016/j.jconrel.2016.05.04427208862

[9] Roney C, Kulkarni P, Arora V, et al. Targeted nanoparticles for drug delivery through the blood-brain barrier for Alzheimer’s disease. *J Control Release*. 2005;108(2–3):193–214. doi:10.1016/j.jconrel.2005.07.02416246446

[10] Tsou YH, Zhang XQ, Zhu H, Syed S, Xu X. Drug delivery to the brain across the blood-brain barrier using nanomaterials. *Small*. 2017;13(43). doi:10.1002/smll.20170192129045030

[11] Zhou Y, Peng Z, Seven ES, Leblanc RM. Crossing the blood-brain barrier with nanoparticles. *J Control Release*. 2018;28(270):290–303. doi:10.1016/j.jconrel.2017.12.01529269142

[12] Ding S, Khan AI, Cai X, et al. Overcoming blood-brain barrier transport: advances in nanoparticle-based drug delivery strategies. *Mater Today*. 2020;37:112–125. doi:10.1016/j.mattod.2020.02.001PMC757513833093794

[13] Jantas D, Warszyński P, Lasoń W. Carnosic acid shows higher neuroprotective efficiency than edaravone or ebselen in in vitro models of neuronal cell damage. *Molecules*. 2023;29(1):119. doi:10.3390/molecules2901011938202702 PMC10779571

[14] Aruoma OI, Halliwell B, Aeschbach R, Löligers J. Antioxidant and pro-oxidant properties of active rosemary constituents: carnosol and carnosic acid. *Xenobiotica*. 1992;22(2):257–268. doi:10.3109/004982592090466241378672

[15] Hou CW, Lin YT, Chen YL, et al. Neuroprotective effects of carnosic acid on neuronal cells under ischemic and hypoxic stress. *Nutr Neurosci*. 2012;15(6):257–263. doi:10.1179/1476830512Y.000000002122687582

[16] Jordán MJ, Lax V, Rota MC, Lorán S, Sotomayor JA. Relevance of carnosic acid, carnosol, and rosmarinic acid concentrations in the in vitro antioxidant and antimicrobial activities of Rosmarinus officinalis (L.) methanolic extracts. *J Agric Food Chem*. 2012;60(38):9603–9608. doi:10.1021/jf302881t22957812

The article "Chitosan-Based Nanocapsules as a Delivery System of Hydrophobic Carnosic Acid, A Model Neuroprotective Drug" was published in 2024. Journal: Nanotechnol Sci Appl.

[17] Oh J, Yu T, Choi SJ, et al. Syk/Src pathway-targeted inhibition of skin inflammatory responses by carnosic acid. *Mediators Inflamm*. 2012;2012:1–13. doi:10.1155/2012/781375PMC333768122577255

[18] Yesil-Celiktas O, Sevimli C, Bedir E, Vardar-Sukan F. Inhibitory effects of rosemary extracts, carnosic acid and rosmarinic acid on the growth of various human cancer cell lines. *Plant Foods Human Nutr*. 2010;65(2):158–163. doi:10.1007/s11130-010-0166-420449663

[19] Birtić S, Dussort P, Pierre FX, Bily AC, Roller M. Carnosic acid. *Phytochemistry*. 2015;115(1):9–19. doi:10.1016/j.phytochem.2014.12.02625639596

[20] Razboršek MI, Ivanović M. Stability studies and determination of carnosic acid and its oxidative degradation products by gas chromatography–mass spectrometry. *Int J Mass Spectrom*. 2016;407:29–39. doi:10.1016/j.ijms.2016.07.002

[21] Szafraniec J, Odrobinska J, Lachowicz D, Kania G, Zapotoczny S. Chitosan-based nanocapsules of core-shell architecture. *Polimery*. 2017;62(7/8):509–515. doi:10.14314/polimery.2017.509

[22] Gumieniczek-Chłopek E, Odrobinska J, Straczek T, Radziszewska A, Zapotoczny S, Kapusta C. Hydrophobically coated superparamagnetic iron oxides nanoparticles incorporated into polymer-based nanocapsules dispersed in water. *Materials*. 2020;13(5):1219. doi:10.3390/ma1305121932182749 PMC7085046

[23] Janik-Hazuka M, Szafraniec-Szczęsny J, Kamiński K, Odrobińska J, Zapotoczny S. Uptake and in vitro anticancer activity of oleic acid delivered in nanocapsules stabilized by amphiphilic derivatives of hyaluronic acid and chitosan. *Int J Biol Macromol*. 2020;1(164):2000–2009. doi:10.1016/j.ijbiomac.2020.07.28832781133

[24] Bulwan M, Zapotoczny S, Nowakowska M. Robust “one-component” chitosan-based ultrathin films fabricated using layer-by-layer technique. *Soft Matter*. 2009;5(23):4726–4732. doi:10.1039/b909355a

[25] Szafraniec J, Błazejczyk A, Kus E, et al. Robust oil-core nanocapsules with hyaluronate-based shells as promising nanovehicles for lipophilic compounds. *Nanoscale*. 2017;9(47):18867–18880. doi:10.1039/c7nr05851a29177344

[26] Odrobińska J, Gumieniczek-Chłopek E, Szuwarzyński M, et al. Magnetically navigated core-shell polymer capsules as nanoreactors loadable at the oil/water interface. *ACS Appl Mater Interfaces*. 2019;11(11):10905–10913. doi:10.1021/acsami.8b2269030810298

[27] Leskiewicz M, Jantas D, Regulska M, et al. Antidepressants attenuate the dexamethasone-induced decrease in viability and proliferation of human neuroblastoma SH-SY5Y cells: a involvement of extracellular regulated kinase (ERK1/2). *Neurochem Int*. 2013;63(5):354–362. doi:10.1016/j.neuint.2013.07.00723906970

The article "Chitosan-Based Nanocapsules as a Delivery System of Hydrophobic Carnosic Acid, A Model Neuroprotective Drug" was published in 2024. Journal: Nanotechnol Sci Appl.

[28] Sadat SMA, Jahan ST, Haddadi A. Effects of size and surface charge of polymeric nanoparticles on in vitro and in vivo applications. *J Biomater Nanobiotechnol*. 2016;07(02):91–108. doi:10.4236/jbnb.2016.72011

[29] Schaeublin NM, Braydich-Stolle LK, Schrand AM, et al. Surface charge of gold nanoparticles mediates mechanism of toxicity. *Nanoscale*. 2011;3(2):410–420. doi:10.1039/c0nr00478b21229159

[30] Liu Y, Li W, Lao F, et al. Intracellular dynamics of cationic and anionic polystyrene nanoparticles without direct interaction with mitotic spindle and chromosomes. *Biomaterials*. 2011;32(32):8291–8303. doi:10.1016/j.biomaterials.2011.07.03721810539

[31] Fröhlich E. The role of surface charge in cellular uptake and cytotoxicity of medical nanoparticles. *Int J Nanomedicine*. 2012;7:5577–5591. doi:10.2147/IJN.S3611123144561 PMC3493258

[32] Hühn D, Kantner K, Geidel C, et al. Polymer-coated nanoparticles interacting with proteins and cells: focusing on the sign of the net charge. *ACS Nano*. 2013;7(4):3253–3263. doi:10.1021/nn305929523566380

[33] Tahara K, Sakai T, Yamamoto H, Takeuchi H, Hirashima N, Kawashima Y. Improved cellular uptake of chitosan-modified PLGA nanospheres by A549 cells. *Int J Pharm*. 2009;382(1–2):198–204. doi:10.1016/j.ijpharm.2009.07.02319646519

[34] Aibani N, Rai R, Patel P, Cuddihy G, Wasan EK. Chitosan nanoparticles at the biological interface: implications for drug delivery. *Pharmaceutics*. 2021;13(10):1686. doi:10.3390/pharmaceutics1310168634683979 PMC8540112

[35] Foged C, Brodin B, Frokjaer S, Sundblad A. Particle size and surface charge affect particle uptake by human dendritic cells in an in vitro model. *Int J Pharm*. 2005;298(2):315–322. doi:10.1016/j.ijpharm.2005.03.03515961266

[36] Nafee N, Schneider M, Schaefer UF, Lehr CM. Relevance of the colloidal stability of chitosan/PLGA nanoparticles on their cytotoxicity profile. *Int J Pharm*. 2009;381(2):130–139. doi:10.1016/j.ijpharm.2009.04.04919450671

[37] Zhao F, Zhao Y, Liu Y, Chang X, Chen C, Zhao Y. Cellular uptake, intracellular trafficking, and cytotoxicity of nanomaterials. *Small*. 2011;7(10):1322–1337. doi:10.1002/smll.20110000121520409

[38] Dash BC, Réthoré G, Monaghan M, Fitzgerald K, Gallagher W, Pandit A. The influence of size and charge of chitosan/polyglutamic acid hollow spheres on cellular internalization, viability and blood compatibility. *Biomaterials*. 2010;31(32):8188–8197. doi:10.1016/j.biomaterials.2010.07.06720701967

[39] El Badawy AM, Silva RG, Morris B, Scheckel KG, Suidan MT, Tolaymat TM. Surface charge-dependent toxicity of silver nanoparticles. *Environ Sci Technol*. 2011;45(1):283–287. doi:10.1021/es103418821133412

The article "Chitosan-Based Nanocapsules as a Delivery System of Hydrophobic Carnosic Acid, A Model Neuroprotective Drug" was published in 2024. Journal: Nanotechnol Sci Appl.

[40] Schauer R. Sialic acids as regulators of molecular and cellular interactions. *Curr Opin Struct Biol*. 2009;19(5):507–514. doi:10.1016/j.sbi.2009.06.00319699080 PMC7127376

[41] Kettler K, Veltman K, van de Meent D, van Wezel A, Hendriks AJ. Cellular uptake of nanoparticles as determined by particle properties, experimental conditions, and cell type. *Environ Toxicol Chem*. 2014;33(3):481–492. doi:10.1002/etc.247024273100

[42] Gosens I, Costa PM, Olsson M, et al. Pulmonary toxicity and gene expression changes after short-term inhalation exposure to surface-modified copper oxide nanoparticles. *NanoImpact*. 2021;22:100313. doi:10.1016/j.impact.2021.10031335559970

[43] Awashra M, Młynarz P. The toxicity of nanoparticles and their interaction with cells: an in vitro metabolomic perspective. *Nanoscale Adv*. 2023;5(10):2674–2723. doi:10.1039/d2na00534d37205285 PMC10186990

[44] Oh I, Min HS, Li L, et al. Cancer cell-specific photoactivity of pheophorbide a-glycol chitosan nanoparticles for photodynamic therapy in tumor-bearing mice. *Biomaterials*. 2013;34(27):6454–6463. doi:10.1016/j.biomaterials.2013.05.01723755832

[45] Farshbaf M, Davaran S, Zarebkohan A, Annabi N, Akbarzadeh A, Salehi R. Significant role of cationic polymers in drug delivery systems. *Artif Cells Nanomed Biotechnol*. 2018;46(8):1872–1891. doi:10.1080/21691401.2017.139534429103306

[46] Chen JH, Ou HP, Lin CY, et al. Carnosic acid prevents 6-hydroxydopamine-induced cell death in SH-SY5Y cells via mediation of glutathione synthesis. *Chem Res Toxicol*. 2012;25(9):1893–1901. doi:10.1021/tx300171u22894569

[47] Wu CR, Tsai CW, Chang SW, Lin CY, Huang LC, Tsai CW. Carnosic acid protects against 6-hydroxydopamine-induced neurotoxicity in in vivo and in vitro model of Parkinson’s disease: involvement of antioxidative enzymes induction. *Chem Biol Interact*. 2015;5(225):40–46. doi:10.1016/j.cbi.2014.11.01125446857

[48] de Oliveira MR, Ferreira GC, Schuck PF, Dal Bosco SM. Role for the PI3K/Akt/Nrf2 signaling pathway in the protective effects of carnosic acid against methylglyoxal-induced neurotoxicity in SH-SY5Y neuroblastoma cells. *Chem Biol Interact*. 2015;242:396–406. doi:10.1016/j.cbi.2015.11.00326577515

[49] de Oliveira MR, Peres A, Ferreira GC, Schuck PF, Bosco SM. Carnosic acid affords mitochondrial protection in chlorpyrifos-treated Sh-Sy5y cells. *Neurotox Res*. 2016;30(3):367–379. doi:10.1007/s12640-016-9620-x27083155

[50] Liu J, Su H, Qu QM. Carnosic acid prevents beta-amyloid-induced injury in human neuroblastoma SH-SY5Y cells via the induction of autophagy. *Neurochem Res*. 2016;41(9):2311–2323. doi:10.1007/s11064-016-1945-627168327

